# The epidemiology and chemotherapeutic approaches to the control of urinary schistosomiasis in school-age children (SAC): a systematic review

This article has been retracted.

**DOI:** 10.1186/s12879-018-3647-y

**Published:** 2019-01-18

**Authors:** Tolulope Ebenezer Atalabi, Taiwo Oluwakemi Adubi

**Affiliations:** 1 Department of Biological Sciences, Federal University, Dutsin-Ma, Km 65, P.M.B. 5001, Dutsin-Ma, Katsina State Nigeria; 2 Department of Biological Sciences and Biotechnology, College of Pure and Applied Sciences, Caleb University, Imota, Lagos State Nigeria

**Keywords:** Prevalence, Control, Urinary, Schistosomiasis, School, Children

## Abstract

**Background:**

Human schistosomiases are acute and chronic infectious diseases of poverty. Currently, epidemiological data of urinary schistosomiasis (US) in school-age children (SAC) and adults are often reported together making it difficult to ascertain the true status of the disease. Based on this premise, we set out to carry out this review.

**Method:**

To achieve this aim, we carried out a computer-aided search of PubMed, Web of Science, Science Direct, African Journals OnLine (AJOL) and the database of World Health Organization. However, the information obtained from these sources was supplemented with additional literatures from Mendeley, Research Gate, and Google.

**Results:**

The search yielded 183 literatures of which 93 full text research, review and online articles were deemed fit for inclusion. Our key findings showed that: (1) of all World Health Organization (WHO) Regions, Africa is the most endemic zone for US, with Kenya and Senegal recording the highest prevalence and mean intensity respectively; (2) SAC within the range of 5–16 years contribute most significantly to the transmission cycle of US globally; (3) gender is a factor to watch out for, with male often recording the highest prevalence and intensity of infection; (4) contact with open, potentially infested water sources contribute significantly to transmission; (5) parental factors (occupation and education status) predispose SAC to US; (6) economic *vis a vis* ecological factors play a key role in infection transmission; and (7) in the last decade, a treatment coverage of 45% was never achieved globally for SAC or non-SAC treatment category for urinary schistosomiasis.

**Conclusion:**

In view of the WHO strategic plan to eliminate schistosomiasis by 2020 and the findings from this review, it is obvious that this goal, in the face of realities, might not be achieved. It is imperative that annual control programmes be scaled up marginally, particularly in the African region of WHO. While US-based researches should be sponsored at the grass-root level to unveil hidden endemic foci, adequate facilities for Water, Sanitation, and Hygiene (WASH) should be put in place in all schools globally.

## Background

Human schistosomiases are acute and chronic infectious diseases associated with abject poverty in 78 low and middle-income countries in the sub-tropical and tropical parts of the world where there is negligible access to potable water and adequate sanitation. The agents of etiology of these diseases are “blood-thirsty” digenetic trematodes in the genus *Schistosoma* [1, 2].

Freshwater gastropod snails in the genus *Bulinus* are suitable intermediate hosts to *Schistosoma haematobium* which causes urinary schistosomiasis. The transmission gap of the disease is bridged when people come into contact with unwholesome water sources [3–5] infested with the cercariae (infective larval form) which mechanically penetrates the skin of their human definitive hosts. A transmission cycle is consolidated when infected humans, due to lack of modern waste disposal facilities, indiscriminately pass urine-infested eggs in close proximity to water bodies where they hatch into larval form (called miracidia) which infect *Bulinus*. In humans, cercariae undergo series of larval migration before maturing into adults which migrate to the veins of the urinary tract where gravid females lay a large number of eggs which are responsible for the various signs, symptoms and morbidity associated with the disease. The classical sign of urinary schistosomiasis is haematuria, a term coined to describe the presence of blood in urine. Genital schistosomiais causes pathological damage in both sexes, with females being more at risk of contracting Human Immuno-Deficiency Virus (HIV) [6, 7].

Nonetheless, a review of the burden of schistosomiasis has shown that over 200, 000 people die from the complications due to the disease in Sub-Saharan Africa (SSA) annually while children suffer anaemia, stunted growth [8, 9], urinary tract damage [10] and reduced mental ability to cope with academics. In advanced cases, hydronephrosis, [11] ureteral and bladder fibrosis/cancer commonly occur [6].

As a follow up to the 2001 World Health Assembly resolution WHA54.19, many endemic countries in Africa launched national control programmes largely based on preventive chemotherapeutic intervention with praziquantel (PZQ) targeting at least 75% of school-age children-SAC (5─14 years old) and adults at risk of schistosomiasis [12, 13] by 2010. This resolution aligns properly with earlier report that SAC, adolescent and young adults usually recorded the highest prevalence and intensities of schistosomiasis [14]. Meanwhile, the guideline of World Health Organization required that treatment of SAC (enrolled and not enrolled) be done: once every year for high-risk communities, once every two years for moderate-risk communities and twice during their Primary School Age in low-risk communities [13, 15].

Currently, epidemiological data on prevalence, intensity and control of US in SAC and adults are often reported together, thus making information peculiar to SAC to be insufficient in the literature. The implication of this is that it is difficult to ascertain the epidemiological status of the disease in this group to enhance the success of control programmes targeting this group. Based on this premise, the aim of this review article was to study the epidemiology and chemotherapeutic strategies to the control of US in SAC.

## Methods

### Search strategy

We carried out a computer-aided search of PubMed, Web of Science, Science Direct, African Journals OnLine (AJOL) and the database of World Health Organization (WHO). However, the information obtained from these sources was supplemented with additional literatures from Mendeley, Research Gate, and Google. The searches were performed independently by the authors using the key words: “urinary/urinary schistosomiasis” in combination with “prevalence”, “intensity”, “morbidity”, “control/praziquantel”, “school” and “children”.

### Selection criteria

Literatures that address prevalence, intensity, morbidity, indicators or risk factors as well as the control of US, without restriction to year of publication, were included in this review article. Besides, such papers addressed school children specifically. The implication of this is that articles exclusively addressing intestinal schistosomiasis or other Neglected Tropical Diseases were not considered eligible for inclusion.

### Analysis and presentation of data

The secondary data presented in this manuscript were manually extracted from the articles included in this review paper. Data imported into Microsoft Excel Spreadsheet were used to generate Bar Charts.

## Results

### The search

The search yielded 183 literatures. After proper scrutiny of the retrieved literatures, 93 full text research, review and online articles were deemed fit for inclusion. Consequently, this review is a product of the findings from these articles. The flow chart in Fig. 1 shows the result of our search.

**Fig. 1:** Flowchart of the article search and selection process

### Characteristics of the included articles

Of the 93 literatures included in this review, majority, 46 (49.46%), were products of researches/reviews carried out in African WHO Region, with Nigeria recording the second largest number of articles, 19 (20.43%). Switzerland in European Region, however, accounted for the largest, 22 (23.66%), which were all technical reports/review articles (see Table 1).

**Table 1:** Descriptive statistics (estimates) of the features of the articles included in the systematic review

Variable	Category A	Category B (who region)	Number of articles	%
Countries	Nigeria	Africa	19	20.43
	Cameroon	Africa	3	3.23
	Cote d’Ivoire	Africa	1	1.08
	Mali	Africa	1	1.08
	Kenya	Africa	8	8.60
	Senegal	Africa	4	4.30
	United State of America	The Americas	3	3.23
	South Africa	Africa	2	2.15
	Switzerland	Europe	22	23.66
	Netherlands	Europe	1	1.08
	Swaziland	Africa	1	1.08
	United Kingdom	Europe	3	3.23
	Yemen	Eastern Mediterranean	1	1.08
	Malawi	Africa	1	1.08
	Niger	Africa	1	1.08
	Ghana	Africa	1	1.08
	Burkina Faso	Africa	1	1.08
	Zimbabwe	Africa	1	1.08
	Zambia	Africa	1	1.08
	Angola	Africa	1	1.08
	Tanzania	Africa	1	1.08
	Ethiopia	Africa	2	2.15
	Others		14	15.05
Type of Article	Research		61	65.59
	Review		6	6.45
	Technical report		22	23.66
	Online article		4	4.30
*Sample year	1984─1993		4	6.56
	1994─2003		4	6.56
	2004─2017		44	72.13
	Not reported		9	14.75
*Sampling method	Cluster		2	3.28
	Random		19	31.15
	Universal/census		4	6.56
	Stratified		2	3.28
	Not reported		33	54.09
	Fish bowl/ systematic		1	1.64
*Study type	Cross-sectional		40	65.58
	Longitudinal		5	8.19
	Not reported		16	26.23
*Sample size determination	Yes		11	18.03
	Not reported		30	49.18
	Could not be ascertained		20	32.78
*Setting	School		39	63.93
	Community		9	14.75
	Others		13	21.31
*Population area	Rural		37	60.66
	Peri-urban		7	11.48
	Others		17	27.87
**Mode of diagnosis	Microscope only		18	43.90
	Real time PCR Assays + Reagent strip + Test for cSEA + microscopy		1	2.44
	Reagent strip only		1	2.44
	Microscopy and Reagent strip		21	51.22
**Format of intensity	Arithmetic mean only		5	12.19
	Geometric mean only		3	7.32
	WHO categories only		13	31.71
	Geometric+ WHO categories		1	2.44
	Not reported/Not specified		19	46.34

*Only applicable to research articles; **Only applicable to prevalence/ intensity studies on humans; cSEA, Circulating Soluble Egg Antigen

The sampling years reported by the 61 research articles included in this review ranged from 1984 to 2017, with the studies executed between 2004 and 2017 being 11 times more in number than those carried out in each of 1984–1993 and 1994–2003. Sixty-Five point Fifty-Eight percent (40), 63.93% (39), and 60.66% (37) of the studies were cross-sectional in nature, carried out in school settings and rural areas respectively (see Table 1).

However, it is worthy of note that sample size determination, sampling method, and intensity of US were not reported by 49.18% (30), 54.09% (33) and 46.34% (19) of the studies included in this review (see Table 1).

## Prevalence and intensity of urinary schistosomiasis

Data on the prevalence of US in different endemic settings are presented in Table 2 below. In Nigeria, the prevalent rates obtained from 14 research articles with a total sample size of 5675 ranged from 2.07%–78.43%. They showed that 2116 school children were infected, giving an overall prevalence rate of 37.29%. Coincidentally, these articles represent the six (6) geopolitical zones of Nigeria.

**Table 2:** Urine Processing Technique, Prevalence, and intensity of urinary schistosomiasis by country’s subarea

Ref	Country	Subarea	Eggs concentration technique	Sample size	Prevalence (%)	Mean Intensity	Age group (Years)
[45]	Nigeria	Kwara State	Centrifugation	551	35.20	N.R	9─16
[46]	Cameroon	Northern Province	Sedimentation	964	36	N.R	9─17
[47]	Nigeria	Plateau State	Sedimentation	242	2.07	27.8**	5─14
[48]	Nigeria	Kano State	Centrifugation	493	44.20	107.30**	5─16
[49]	Kenya	Migori County	Filtration	1768	8.90	N.R	7─14
[50]	Nigeria	Adamawa State	Centrifugation	232	47.80	8.30**	4─15
[51]	Kenya	Coast Province	Filtration	12,541	41.50	45*	5─19
[52]	Kenya	Coast Province	Filtration	7093	66	20**	5─21
[53]	Senegal	Fatick Region	Filtration	329	73.20	356.1*	5─15
[54]	Nigeria	Katsina State	Centrifugation	611	21.11	26.98**	10─15
[55]	Kenya	North Coast	Filtration	262	94	N.R	5─12
[56]	Nigeria	Ogun State	Centrifugation	487	57.1	45**	6─14
[57]	Malawi	Chikhwawa district	Centrifugation	1642	14.20	N.R	N.R
[58]	Niger	Tillabery /Tahoua	Filtration	1642	75.40	15.50*	7,8 & 11
[59]	Kenya	Coast Province	Filtration	4031	35	N.R	N.R
[60]	Ghana	Brong Ahafo Region	Centrifugation	100	50	N.R	6─15
[61]	Senegal	Fatick Region	Filtration	682	57.6	N.R	5─15
[62]	Cameroon	Magba Region	Filtration	382	41.10	154.7**	7─14
[63]	Senegal	Fatick Region	Filtration	210	57.6	185*	7─15
[64]	Nigeria	Lagos State	Sedimentation	102	78.43	N.R	5─15
[65]	Burkina Faso	Ouagadougou	Filtration	3514	8.76	6**	7─11
[66]	Zimbabwe	Chikwaka Communal Land	N.R	551	60	N.R	9─16
[67]	Nigeria	Katsina State	Centrifugation	436	27.98	35.29**	12─17
[68]	Zambia	Lusaka Province	Filtration	2040	9.60	31.40**	6─15
[69]	Nigeria	Ogun State	Centrifugation	187	64.7	0.95*	5─15
[70]	Kenya	Coast Province	Filtration	114	22.8	N.R	N.R
[71]	Angola	Cubal District	N.R	785	61.80	N.R	9─10
[72]	Yemen	Taiz, Ibb, Dhamar, Sana’a and Hodiedah Provinces	Filtration	400	23.80	N.R	†
[73]	Nigeria	Kaduna State	Centrifugation	505	12.30	2.69**	4─15
[74]	Nigeria	Rivers State	Sedimentation	130	23.10	N.R	5─16
[75]	Ethiopia	Gambella Regional State	Filtration	304	35.90	8.76**	7─14
[76]	Ethiopia	Almost all regions	Filtration	99,726	0.20	N.R	10─15
[77]	Nigeria	Adamawa State	Centrifugation	346	32.40	N.R	5─15
[78]	Nigeria	Taraba State	Filtration	1153	53.08	N.R	6─15
[79]	Nigeria	Cross River State	Filtration	200	21	N.R	5─15
TOTAL				144,755			

*Geometric Mean Intensity; N. R, Not reported; **Arithmetic Mean Intensity; † Not clearly defined

However, six studies from Kenya reported that of the 25, 809 respondents sampled, 11,728 were infected with the infective stage of *S. haematobium*, giving a prevalence rate of 45.44%. The prevalence of US obtained from Kenya-based literatures ranged from 8.90%–94%.

Moreover, two Ethiopia-based research articles retrieved showed that of the 100,030 respondents examined, 310 tested positive for US, resulting in a prevalence rate of 0.31%.

In Cameroon, out of the 1346 school children interviewed and examined as reported by two articles, 446 were found to be suffering from the menace of US, giving a prevalence rate of 33.14%.

Furthermore, a prevalence of 67.16% was computed from a total sample size of 539 reported by two papers which showed that 362 school children were infected.

Finally, each research paper obtained from Malawi, Niger, Ghana, Burkina Faso, Yemen, Zimbabwe, Zambia and Angola reported prevalence rates (sample size) of: 14.20% (1642), 75.40% (1642), 50% (100), 8.76% (3514), 23.80% (400), 60% (551), 9.60% (2040) and 61.80% (785) respectively.

Table 2 also presents the extracted data on the intensity of US. It is obvious that only 17 research articles (48.57%) reported the intensity of infection due to the disease in question. Of this figure, 12 (70.59%) presented mean intensity of infection as Arithmetic Mean while only 5 (29.41%) presented it as Geometric Mean.

By Arithmetic format of reporting mean intensity, the highest value, 154.7 eggs per 10 ml of urine sample, was reported in a survey carried out in Magba Region, Cameroon while the runner up value, 107.30 eggs per 10 ml of urine sample, was reported from Kano State, Nigeria. The overall highest mean intensity of infection was reported in Fatick Region, Senegal as a Geometric Mean Intensity of 356.1 eggs per 10 ml of urine sample. The same location recorded the second highest mean egg count of 185 eggs per 10 ml of urine sample.

As it stands, Kenya has the highest prevalence while Senegal has the highest mean intensity of infection with US among SAC.

Of the 41 research articles included in this review paper, 35 reported a total number of 144,755 participants with prevalence/intensity records. As far as *S. haematobium* egg concentration technique was concerned, 11, 18 and 4 articles recorded centrifugation, filtration, and sedimentation as means of preparing sample for viewing under the microscope. However, 2 articles from Angola and Zimbabwe did not report technique of egg concentration.

## Risk factors of urinary schistosomiasis in school children

Table 3 presents the factors that are considered pertinent to the transmission of US in school children. Findings from this review reveal that SAC within the range of 5–16 years of age were consistently and unanimously reported as the group with the highest prevalence and association with US.

**Table 3:** Risk factors of urinary schistosomiasis peculiar to school children

Risk factor	Category	References
Age	7─9	[62]
	5─10	[79]
	10─12	[55]
	12─14	[56]
	11─15	[53]
	5─15	[69]
	6─15	[78]
	13─16	[74]
Gender	Male	[49, 53, 54, 62, 63, 65, 67, 75, 78–80]
	Female	[64, 73, 74]
Recreational activities	Swimming/play in shallow water	[54, 73]
Water sourcing for domestic use	*Unwholesome water sources	[54, 62, 67, 72, 73, 81]
Parental occupation/Farm-related activities	Farming	[54, 57, 73, 75]
	Fishing	[54, 57, 62, 67, 73]
	Brown collar jobs	[54, 67]
	House wives	[54]
	Irrigation	[20]
Parental educational status	Illiteracy	[72, 73]
Proximity of residence to infested water		[71, 72, 81]
Altitude	Valley	[68]
Lack of sewage disposal facilities	Toilet	[72]
Changing global climate		[20]

*Rivers, streams, ponds, and dams

By the findings in this review paper, gender played a significant role in the transmission of US, with males recording higher prevalence of infection and significant association more often over their female counterparts.

Water-related factors like swimming, playing in shallow waters, fetching water for domestic uses in open and potentially infested water bodies like lakes, rivers, ponds, streams, etc. *vis a vis* proximity of residence to sources of unwholesome water sources have all been reported by researchers as key factors in the transmission of the disease.

In addition, parental factors such as educational and occupational status have been reported by researchers from various endemic settings of US.

Finally, economic and ecological factors like lack of sewage disposal facilities and climate change were reported as determinant factors of the disease.

## Pathology and morbidity markers of urinary schistosomiasis

Table 4 presents the pathological consequences and morbidity markers of US by infection phases as reported by the research articles included in this review.

**Table 4:** Reported morbidities by infection phases of urinary schistosomiasis

Infection Phase	Morbidity/Pathological Consequences	References
Larval Invasion	Swimmers itch	[54]
Acute (Maturation)	Eosinophilia	[55]
Chronic (Establishment)	Terminal haematuria	[46, 52, 54–56, 58, 62]
	Proteinuria	[52, 56, 66]
	Dysuria	[46, 54, 62, 66]
	Pseudopolyps	[55, 66]
	Bladder papillomas/lesion	[52, 58]
	Bladder wall calcification	[20]
	Ureteric fibrosis	[52]
	Kidney pyelon dilatation	[55, 58, 66]
	Ureter dilatation	[16, 55, 58]
	Intravesical mass formation	[16]
	Hydronephrosis	[52, 66]
	Genital discharge/itching/burning sensation	[69, 82]
	Genital lesions	[16]
	Genital swelling/lump	[69]

Morbidity markers identified include swimmer’s itch, eosinophilia, terminal haematuria, proteinuria, and dysuria. On a broad note, the morbidities/pathological consequences reported obviously revolve around the urogenital system as shown in Table 4 below. They are majorly associated with the chronic phase of the disease.

Table 5 presents a list of drugs of intervention for US. It shows PZQ as having the highest cure rate and Niridazole as the least.

**Table 5:** Mode of administration, dosage and cure rate of selected drugs for adult *S. haematobium* control

Drugs	Mode of administration	Dosage	Cure rate	References
Antimonials	Intravenous	30 mg/15 kg (12 injections)	82%	[83]
Niridazole	Oral	100 mg/kg	36%	[84]
Metrifonate		10 mg/kg (single)	50.8%	[85]
Praziquantel		40 mg/kg (single)	75%–85%	[86]

Generally, the global population treated for schistosomiasis increased from 2008 to 2016 with the exception of 2011 and 2013 when a decline was experienced (Fig. 2). The same applied to the number of SAC treated as well as their treatment coverage within the same period. The highest distribution coverage for PZQ was achieved in 2016 (see Fig. 3). However, the SAC requiring chemotherapeutic intervention with PZQ kept increasing till 2014 (see Table 6 and Fig. 2).

**Fig. 2:** A clustered column chart showing the population categories of School-Age Children (SAC) treated with Praziquantel between 2008 and 2016 intervention period

**Fig. 3:** A clustered column chart showing the distribution coverage of Praziquantel in the last decade

**Table 6:** Proportion of school-age children requiring treatment and the number treated for schistosomiasis in the past decade

Period of intervention (Year)	Global population treated (Millions)	SAC requiring treatment (Millions)	Reported SAC treated (Millions)	Coverage (%)	References
2008	17.5	N.R	9.6	N.R	[87]
2009	19.6	N.R	10.8	N.R	[88]
2010	33.5	108.9	21.7	19.9	[89]
2011	28.1	111.5	16.5	14.8	[90]
2012	42.1	114.7	29.7	25.9	[91]
2013	39.5	121.2	26.8	22.1	[92]
2014	61.6	123.3	49.2	34.6	[92]
2015	66.5	118.5	53.2	42.2	[32]
2016	89.2	111.2	70.9	53.7	[93]
2017	**	**	**	**	N.A

**Data not available yet; *SAC* School-age Children, *NR* Not reported, *NA* Not applicable

## Discussion

### Results summary

In summary, the overall findings in this review showed that: (1) of all WHO Regions, Africa is the most endemic zone for US, with Kenya and Senegal recording the highest prevalence and mean intensity respectively; (2) SAC within the range of 5–16 years contribute most significantly to the transmission cycle of the disease globally; (3) gender is a factor to watch out for, with male often recording the highest prevalence and intensity of infection; (4) contact with open, potentially infested water sources contribute significantly to its transmission; (5) parental factors (occupation and education status) predispose SAC to US; (6) economic *vis a vis* ecological factors play a key role in infection transmission; and (7) in the last decade, a treatment coverage of 45% was never achieved globally for SAC or non-SAC treatment category for US.

### The need to treat school-age children (SAC)

Meanwhile, schistosomiasis, an infectious disease of poverty, is easily contracted through poor hygiene and play habits of school children. In majority of areas endemic for US, a peak of morbidity is usually observed in school children within age range 7–14 years [16]. On the long run, it prolongs squalor and as a result, blocks cognitive academic performance and normal growth of children. This culminates in suffering and sometimes, death [17]. The extent of morbidity due to US is strongly linked with the intensity and the length of infection period. Because US is more prevalent in SAC, control programme is directed at them so that the duration of heavy infection intensity could be reduced markedly [18, 19].

Unfortunately, as our findings revealed, majority of SAC are from Africa which had previously been reported to have accounted for an estimate of over 85% of all cases of schistosomiasis globally [20]. Therefore, promoting the health of SAC has been an integral part of the programme of WHO, United Nations Educational, Scientific and Cultural Organization (UNESCO), United Nations Children’s Fund (UNICEF), and other international agencies since the 1950s [21]. SAC are a target group for Mass Drug Administration (MDA) since WHO expert committee on schistosomiasis met for the first time 64 years ago [18, 22].

This is ascertained by the projected budget of about USD 116 million for 2009 to 2013 global procurement and delivery of drug to endemic countries by WHO and the UN systems without custom fees and clearance charges due to existing agreements [23, 24]. In Central Nigeria, study on the epidemiology of US in SAC using the WHO paradigm of ≥50% prevalence has been used as a benchmark for the treatment of the disease in adults [25].

### Management strategies of urinary schistosomiasis in SAC and associated challenges

Various strategies have been applied in the control of US. These include indiscriminate mass treatment, active case finding and treatment of particular risk groups such as school-aged children [26]. However, before the advent of PZQ, other drugs effective against different species and stages of development were used (see Table 5). Drugs of intervention for schistosomiasis progressed from antimonial compounds to PZQ which is the drug of choice today [27]. Metrifonate and Hycathone mesylate are effective for the treatment of US. Lucanthone hydrochloride was used from 1948 to mid-sixties. When given a short treatment from 3 to 6 days, it had moderate activity against *S. haematobium*. Niridazole is used against *S. mansoni, S. japonicum* and *S. haematobium* [28]*.* Corticosteroids and anticonvulsants are used to treat katayama fever in order to suppress the hypersensitivity reaction and with PZQ to eliminate the already mature adult. PZQ should be administered with great caution in the case or concurrent neurocysticercosis [29]. The use of Artemisinin derivatives as prophylaxis for acute schistosomiasis, possibly in combination with PZQ, has been investigated. However, Artemisinin use in malaria-endemic areas is not encouraged because of anticipated drug resistance [30].

However, the most rapid and cost-effective way to control morbidity due to schistosomiasis is through a chemotherapeutic intervention with PZQ [31]. PZQ and Albendazole can, however, be administered together safely where there is co-endemicity of schistosomiasis and Soil-Transmitted Helminthiasis (STH) [32]. It is already well known that after chemotherapy, cessation of symptoms is evidenced in the reduction of egg excretion, proteinuria, haematuria, urinary iron loss, leucocyturia, and few remaining schistosomes which cannot multiply [17, 18, 33–36]. Consequently, they pose little or no threat to their hosts. Therefore, control programmes should focus on the achievement of a sharp decline in the intensity of infection [17]. Based on this premise, in 2001, the World Health Assembly adopted resolution 54.19 which set a target for all endemic countries to regularly treat over 75% of all SAC at risk of morbidity due to schistosomiasis and STH by 2010 [37, 38]. It is pertinent to state that the result of this review clearly showed that this aim was not achieved (see Table 6).

Nevertheless, the greatest challenge of MDA is to extend regular drug coverage to reach all the children at risk of morbidity due to infection by helminths [23]. There are two perspectives to this. One, each School-age Child (SAC) treated may not have access to enough PZQ that would clear all the parasites. Two, the distribution coverage may not cater for the whole population of infected SAC. Consequently, symptoms of chronic infection may show up after 5–15 years in children who were partially treated as a result of poor coverage of PZQ [20]. However, the report of a School-Based Treatment carried out in Zanzibar Island, Tanzania, where 8000 pupils were treated showed amazing coverage of 85.2 and 86.9% in Pemba and Unguja Districts respectively [39].

PZQ is not without its adverse reactions like abdominal pain, dizziness, headache, vomiting, diarrhea, round, swollen and itching skin rashes, and fever [40]. These are usually mild and last for 24 h. These are reactions from dying worms.

In addition, studies have shown that false negative results cause infected SAC to escape treatment, leading to chronic condition and if such case occurs after MDA, cure rate may be overestimated and this may be a prelude to drug resistance and further transmission of US [41].

It is hoped that in the nearest future, global schistosomiasis control programmes will receive a boost when the current “evolutionary” process of vaccine-linked chemotherapy culminates in approval by WHO. A good number of these vaccines undergoing preclinical and clinical trials on the field are particularly made for children [42].

### Limitations of the review

This review took articles reported in English into consideration instead of including those reported in other languages. Besides, we noticed that mean intensity of infection with US was either underreported or not reported by some authors of articles included in this review article. Consequently, the report of the mean intensity reported here may not be an accurate reflection of what is obtainable among SAC globally.

## Conclusion

The prevalence rates and intensities of US *vis a vis* its impact on SAC, keep increasing from year to year, leading to increase in the global population requiring chemotherapeutic intervention with PZQ. In view of the WHO strategic ambitious plan to eliminate schistosomiasis by 2020 [43] and the findings from this review stipulating that in the last decade, a PZQ distribution coverage of 45% has never been achieved for SAC, it is obvious that this goal, in the face of realities, might not be achieved just like the strategic plan for 2010. Our view is in agreement with the report that if WHO sustains the current treatment trend, elimination is achievable in 2030 [44]. It is imperative that annual control programmes be scaled up marginally, particularly in the African region of the WHO. While US-based researches should be sponsored at the grass-root level to unveil hidden endemic foci, adequate facilities for Water, Sanitation, and Hygiene (WASH) should be put in place in all schools globally.
